The article "Deep Learning-Based Image Reconstruction for Different Medical Imaging Modalities" was published in 2022. Journal: Comput Math Methods Med.

# Deep Learning-Based Image Reconstruction for Different Medical Imaging Modalities

**DOI:** 10.1155/2022/8750648

**Published:** 2022-06-16

**Authors:** Muhammad Yaqub, Feng Jinchao, Kaleem Arshid, Shahzad Ahmed, Wenqian Zhang, Muhammad Zubair Nawaz, Tariq Mahmood

**Affiliations:** ^1^Beijing Key Laboratory of Computational Intelligence and Intelligent System, Faculty of Information Technology, Beijing University of Technology, Beijing 100124, China; ^2^College of Science and Shanghai Institute of Intelligent Electronics and Systems, Donghua University, 24105 Songjiang District, Shanghai, China; ^3^Division of Science and Technology, University of Education, Lahore, Pakistan

## Abstract

Image reconstruction in magnetic resonance imaging (MRI) and computed tomography (CT) is a mathematical process that generates images at many different angles around the patient. Image reconstruction has a fundamental impact on image quality. In recent years, the literature has focused on deep learning and its applications in medical imaging, particularly image reconstruction. Due to the performance of deep learning models in a wide variety of vision applications, a considerable amount of work has recently been carried out using image reconstruction in medical images. MRI and CT appear as the ultimate scientifically appropriate imaging mode for identifying and diagnosing different diseases in this ascension age of technology. This study demonstrates a number of deep learning image reconstruction approaches and a comprehensive review of the most widely used different databases. We also give the challenges and promising future directions for medical image reconstruction.

## 1. Introduction

The reconstruction of images is an integral part of several systems of visual perception. This includes partitioning several segments or objects [1] with images. Reconstruction of medical images is one of the most basic and essential elements of medical imaging, the main goal of which is to obtain high-quality medical images for clinical use at the lowest cost and risk to patients. The process of image reconstruction can be characterized as a way of importing two-dimensional images into a computer, then improving or exploring the image by transforming it into a form that is more constructive and useful to the human observer. In computer vision and image processing, deep learning has been commonly used to deal with existing images, enhance these images, and generate features from them. Deep learning (DL) approaches have been effectively applied in medical imaging, including computer-aided detection and diagnosis, radionics, and medical image analysis [2, 3]. In a wide variety of applications, deep neural networks are highly effective, often with a higher degree of human efficiency. For example, with the energy usage of popular graphic processing units, making thousands of predictions a day brings with it such a considerable amount of energy. Equally, in terms of the speed deep neural network can deliver and the transmission of NNs with millions of parameters across small band channels, legitimate predictions are often around one hundred meters away. This means that it takes significant changes in all these issues to operate on hardware-related devices, such as smart phones, robots, or vehicles. Compaction and performance have also become a focus of concern in the field of deep learning. The recent increase in deep learning techniques has made it possible for deep models to solve increasingly difficult and complex problems. Convolution neural networks (CNNs) have shown that in all areas of existence, they outperform invariant solutions and sophisticated algorithms for reconstruction. Deep learning has been a huge success, and in particular, data analysis has now become a rising trend [4, 5]. The most important patches in the image are first detected in the proposed system I, and then, a three-hidden-layer convolutional neural network (CNN) is designed and trained for feature extraction and patch classification. The proposed system II uses a two-layer long short-term memory (LSTM) network for classification and a CNN for feature extraction. For image grading, the LSTM network is used to simultaneously consider all patches of an image [6]. Recent advances in efficient computational resources, including cloud computing systems and GPUs, have increased the usage and applicability of deep learning in a variety of disciplines, particularly medical image reconstruction [7].

The article "Deep Learning-Based Image Reconstruction for Different Medical Imaging Modalities" was published in 2022. Journal: Comput Math Methods Med.

The remainder of this work is structured as follows: Section 2 gives an overview of deep learning applications in medical imaging.  Section 2.1 reviews techniques of image reconstruction.  Section 2.9 lists a detailed discussion of widely used databases for medical image reconstruction. The key problems and future directions for image reconstruction are discussed in Section 3. In Section 3.2, we present our review conclusions.

### 1.1. Deep Learning-Based Image Reconstruction

ANNs are the foundation of deep learning techniques [8]. Deep learning gained popularity in 2012, when a DL-based approach dominated a computer vision competition. Furthermore, deep learning approaches have increased their performance since 2010, and by 2015, they have surpassed human accuracy in large-scale image identification problems [6]. Deep learning directly learns from image data, whereas conventional approaches require human involvement for feature extraction [2]. The studies [8–10] provide a more general review of deep learning. They propose a deep feed-forward neural network approach to classify binary microarray datasets [11]. The proposed method is tested against CNS, Colon, Prostate, Leukemia, Ovarian, Lung-Harvard2, Lung Michigan, and Breast cancers using eight standard microarray cancer datasets. According to the study [12], the area of medical imaging reconstruction has gone through three stages of growth, as shown in Table 1.

### 1.2. Medical Image Reconstruction Using Deep Learning on MRI

Deep learning applications in medical image reconstruction have a modest amount of published material. Machine learning, according to scientists, might also be used for medical image reconstruction, as it has been effectively used for image-processing tasks such as classification, segmentation, super-resolution, and edge detection. The primary goal of our research is to conduct a review of the current literature on medical image reconstruction. In [13–15], related research can be found on medical imaging. MRI has revolutionized radiology and medicine since its beginning in the early 1970s [16]. In addition to a high-quality data collection process, image reconstruction is a key step in guaranteeing good MRI image quality. While the first magnetic resonance images were acquired by using an iterative reconstruction algorithm [16] from data resembling radial projections of the imaged specimen, non-Cartesian acquisition and iterative reconstruction techniques were not implemented for several years in clinical MRI, and their use is still very limited today. There are two explanations behind this: First, in the case of homogeneity or gradient waveform imperfections, the fundamental presumption that the measured data is radial representations of the imaged object fails. Second, the practical application is restricted by the long reconstruction times associated with iterative reconstruction algorithms. MRI reconstruction became practical and the image quality acceptable only after the introduction of spin-warp (Cartesian) imagery [17], which made it possible to use the fast Fourier transform (FFT) for image reconstruction. MRI reconstruction was made effective by the *k*-space formalism [18, 19] and the FFT. This susceptibility to multieffects makes MRI scans very resilient but also vulnerable to artefacts. The simple Fourier signal model must be developed to offer the whole physical description underlying image generation in order to produce an artefact-free image or a quantitative map of a tissue or device attribute [20]. The system view of MRI has been presented in Figure 1. This can be achieved by formulating the reconstruction of the image as an inverse problem and applying a suitable algorithm to solve it. MRIs have come a long way over the last 45 years. With the growing computational capacity and the growth of novel reconstruction techniques, we are now able to solve more complex problems in appropriate reconstruction times. The availability of technical facilities as well as the availability and use of medical technology of the European Union (EU) [21] is presented in Figure 2. The medical technology concerns a variety of equipment used for diagnostic imaging, for example, magnetic resonance imaging (MRI) units. While several model-based reconstruction techniques have been developed to solve a specific problem, it is still a challenge to address a complete explanation of the reconstruction measurement process in future works.  Table 2 shows an overview of some of the papers reviewed. Furthermore, we reviewed other modalities including CT, ultrasound, and PET.

The article "Deep Learning-Based Image Reconstruction for Different Medical Imaging Modalities" was published in 2022. Journal: Comput Math Methods Med.

### 1.3. Medical Image Reconstruction Using Deep Learning on CT

In CT, image reconstruction is accomplished by the use of projection data. When the projection data is sufficiently comprehensive, filtered back projection (FBP) techniques generate high-quality images. However, some applications, such as reducing scan time, lowering X-ray radiation, which may expose patients to additional health concerns, and scanning of some lengthy objects with restricted angular range, may result in inadequate projection data, making FBP algorithms ineffective. Iteratives such as total variation- (TV-) based algorithms produce acceptable quality reconstructions from partial projection data; however, certain artefacts arise at the margins of a reconstructed image if the projection data is gathered by a reduced CT-angle. Deep learning methods are currently being utilized to solve these issues [22], including PYRO-NN [23], Learn [24], DEAR [25], GoogLeNet Improved [26], among other deep frameworks for image reconstruction in CT. In contrast to established traditional techniques, a series of other research also reveals exact image reconstruction [27]. These deep learning techniques have been utilized for 2D and 3D reconstruction, reducing noise efficiently, improving spatial resolution, and working more quickly on processor graphics units (GPUs). A summary of articles that use deep learning approaches is provided in Table 3 for image reconstruction in CT.

### 1.4. Deep Learning for Image Reconstruction in Other Imaging Modalities

Deep learning approaches have been employed to reconstruct images in different imaging modalities including ultrasound, PET, optical microscopy [28], fluorescence microscopy [29], electromagnetic tomography (EMT) [30], photoacoustic tomography (PAT) [31], diffuse optical tomography (DOT), monocular colonoscopy [32], stochastic microstructure reconstruction [33], holographic image reconstruction [34], reconstruction of neural volumes [35], tomographic 3D reconstruction of a single-molecule structure [36], neutron tomography [22], coherent imaging systems, and integration of deep and transfer learning in imaging. A summary of articles that use deep learning approaches is provided in Table 4 for image reconstruction in other imaging modalities. Conventional image reconstruction method flow chart is shown in Figure 3.

The article "Deep Learning-Based Image Reconstruction for Different Medical Imaging Modalities" was published in 2022. Journal: Comput Math Methods Med.

## 2. Overview of Traditional Image Reconstruction Techniques

Image reconstruction, in general, is an inverse problem that assists in the recovery of the original ideal image from a supplied inferior version. Image reconstruction is defined as a method of inputting two-dimensional pictures into a computer, then enhancing or exploring the image by changing it into a more constructive and usable shape for the human viewer. Analytical reconstruction and iterative reconstruction are the two main types of reconstruction approaches (IR). In the clinical use of magnetic resonance imaging, image reconstruction plays a crucial role. The role of image reconstruction is to convert the acquired *k*-space data to images that can be interpreted clinically. It is necessary to develop common tools and vocabulary to describe the consistency of the reconstructed image before explaining particular image restoration techniques and the signal processing steps they employ. The concept image quality is not intended to mean that one image is better than another. Here, it is widely used to describe certain characteristics that differentiate between one image reconstruction product and another. Techniques used in medical reconstruction, their strengths, and limitations are presented in Table 1. There are many ways in which it is possible to explain image reconstruction results. A strong noise image denoising method based on improved K-SVD and atom optimization is presented. The proposed method includes sparse coding based on correlation coefficient matching and iterative stopping criteria of an OMP algorithm based on a weak selection iterative threshold strategy in dictionary training [45], in addition to image feature extraction and noise atom suppression. Image reconstruction is used in a wide range of industries and activities in the real world. Reconstruction enables us to obtain insight into qualitative properties of the item that are impossible to discern from a single plane of sight, such as volume and the object's relative location to other objects in the scene. Reconstruction techniques can be used in cardiology, art analysis and restoration, film, television, phenotype analysis and criminal investigations, game graphics, and design.

The article "Deep Learning-Based Image Reconstruction for Different Medical Imaging Modalities" was published in 2022. Journal: Comput Math Methods Med.

### 2.1. Iterative Reconstruction (IR)

In image restoration, there are essentially two approaches: iterative reconstruction and analytical reconstruction. The restoration question in the iterative method is limited to calculating a finite number of image values from a finite number of measurements. Major IR algorithms are compared on different parameters in Table 5. Iterative reversal appears to require more computing resources, but the procurement process can deal with more complicated models.

### 2.2. Algebraic Reconstruction Technique (ART)

ART is a widely recognized iterative approach used for medical image reconstruction to solve equations in the linear system.

(1) $$\begin{array}{c} P_{1}=W_{31}f_{1}+W_{31}f_{1}+W_{31}f_{1}+\cdots +W_{31}f_{1},\\ P_{1}=W_{31}f_{1}+W_{31}f_{1}+W_{31}f_{1}+\cdots +W_{31}f_{1},\\ P_{1}=W_{31}f_{1}+W_{31}f_{1}+W_{31}f_{1}+\cdots +W_{31}f_{1}. \end{array}$$

Equation (1) is related to multilevel thresholding. ART updates the projection values from the projection in Equation (2) and applies a correction factor to determine the pixel value at every *j*-position as defined in Equation (3).

(2) $$\begin{array}{c} P_{I}=\overset{N}{\underset{I=1}{\sum }}W_{I}lf_{i}, \end{array}$$

(3) $$\begin{array}{c} f_{j}^{k=1}=f_{j}^{k}+\frac{p_{i}-\sum_{i=1}^{N}f_{l}^{k}W_{i}l}{\sum_{i=1}^{N}W_{il}^{2}}, \end{array}$$

where *p*_*i*_ is the measured effect projection info, *f*_*j*_ specifies a value on pixels at the *j*-position, *w*_*ij*_ is the *j*_*th*_ pixel weighted ratio that the *i*_*th*_ ray moves around, and *k* is the number of iterations.

### 2.3. Simultaneous Reconstruction Technique (SIRT)

It is believed that SIRT (Simultaneous Iterative Reconstruction Technique) would recreate incorrect acquisition data containing any noise for a reconstructed picture of reasonable quality. SIRT, though, is very slow to reconstruct an image because it takes a lot of time to achieve a sufficiently high precision image during iteration. In addition, the SIRT creates a distorted smoothing effect [62].

### 2.4. Simultaneous Algebraic Reconstruction Technique (SART)

SART, which makes full use of the combination of ART and SIRT algorithms, has been proposed as an upgrade to the ART and SIRT algorithms [62]. ART is a quick convergence operation, whereas SIRT produces an image of high quality, so SART is supposed to have certain useful characteristics. As expressed below in Equation (4), smoothing the noise on core SART is defined as follows:

(4) $$\begin{array}{c} f_{j}^{k=1}=f_{j}^{k}+\lambda \frac{1}{\sum i\varepsilon l\theta }\cdot \sum \cdot \frac{p_{i}-\sum_{i=1}^{N}f_{l}^{k}W_{i}l}{\sum_{i=1}^{N}W_{il}^{2}}\;W_{ij}. \end{array}$$

The article "Deep Learning-Based Image Reconstruction for Different Medical Imaging Modalities" was published in 2022. Journal: Comput Math Methods Med.

### 2.5. Conjugate Gradient (CG)

The algorithm for the gradient descent is designed to prevent the fluctuations. The first iteration is the same as the climb of the highest gradient. The algorithm begins to travel in the context of the highest gradient and, once a maximum is reached, proceeds to move along the same axis. For effective cohesion, several iterations are involved which always leads to a zigzag line. In the subsequent iterations, indeed, the algorithm tends to step in a direction in which the gradient stays the same in the prior direction. In these prior directions, the idea is to remove the need of fresh optimization. We let the previous path be *d*_old_ and the Hessian matrix be *H*. The new path *d*_new_ is now expected to be such that the gradient along *d*_old_ does not change. The gradient would change to *Hd*_new_ when heading in the direction of *d*_new_. Requiring zero for the resulting adjustment to *d*_old_ yields the following situation:

(5) $$\begin{array}{c} \;d_{\text{old}}Hd_{\text{new}}=0. \end{array}$$

### 2.6. Maximum Likelihood Expectation Maximization (MLEM)

The expectation-maximization (EM) algorithm is based on the maximum-likelihood (ML) technique for reconstruction which has a strong theoretical base, is easy to implement, and has proven to be more resilient than filtered back projection (FBP) against noise and systemic anomalies in the data and device matrix. As a result, it is commonly employed in image reconstruction in positron emission tomography (PET) and single photon emission tomography (SPECT) [63].

(6) $$\begin{array}{c} X_{i}^{\left(k+1\right)}=\frac{X_{i}^{\left(k\right)}}{\sum jA_{ji}W_{j}}\underset{j}{\sum }A_{ji}\left(\;\frac{P_{j}}{\sum nA_{jn}X_{i}^{\left(k\right)}}\right), \end{array}$$

where *X*_*i*_^(*k* + 1)^ at the *k*_th_ iteration is the *i*_th_ image pixel, *p*_*j*_ is the measurement value of the *j*th line-integral (ray-sum), and *A*_*ji*_ is the addition of the *i*_th_ image pixel to the measurement of the *j*_th_. The summation over the *n* index is the projector, and the back projector is the summation over the *j* index.

### 2.7. Ordered Subset Expectation Maximization (OSEM)

The ordered subset expectation maximization (OSEM) approach in mathematical optimization is an iterative method that is used in computed tomography. In medical imaging, positron emission tomography, single photon emission computed tomography, and X-ray computed tomography all use the OSEM technique. The OSEM methodology is linked to the expectation maximisation (EM) mechanism in stats. The OSEM mechanism is also linked to FBP strategies. For the OSEM algorithm, the primary upgrade equation is explained by [64].

(7) $$\begin{array}{c} f_{j}^{n,b}=\frac{f_{j}^{n,b-1}}{\sum i\varepsilon s_{b}\;H_{ij}}\cdot \sum i\varepsilon s_{b}\;\frac{p_{i}}{\sum k\;H_{ik}\;f_{i}^{n,b-1}+a_{i}}, \end{array}$$

where the image under reconstruction is *f*, the voxel indices are *j* and *k*, the iteration number is *n*, the subset number is *b*, the subset *b* is *S*_*b*_, the system matrix is *H*, the LOR calculation is *p*, and the scatter and random corrections are models.

The article "Deep Learning-Based Image Reconstruction for Different Medical Imaging Modalities" was published in 2022. Journal: Comput Math Methods Med.

### 2.8. Maximum A Posteriori (MAP)

The principal problems associated with ML algorithms are alleviated by MAP techniques. Next, there are clearer MAP reconstructions than their ML equivalents. Second, with more iterations, iterated MAP estimates appear to hit a point at which they change very little, suggesting estimated convergence [65]. MAP restoration efficiently helped smooth noise and strengthen convergence, with some drawbacks as well. Second, performance can be strongly dependent on parameter selection. Unfortunately, as may be done for post reconstruction filters, it is not effective to use a trial-and-error strategy for parameter collection, since a complete iterative reconstruction should be conducted to test the response from one range of constraints. Second, the loss of image characteristics or, in some situations, the development of spurious characteristics may result from unnecessary smoothing using Gibbs priors. This is a representation of the fact that, in return for reduced noise variation, the MAP estimator introduces some bias to the ML problem. Finally, smoothing properties that are somewhat different from traditional Fourier domain filters used in nuclear medicine are implemented by MAP algorithms, so they can be important for doctors to first interpret.

### 2.9. Analytical Reconstruction

The foundation of the analytical approach is mathematical inversion, offering effective, noniterative algorithms for reconstruction. Through reconstruction based on data by modelling the projection as a line integral form, you may reassemble the image.

### 2.10. Central Slice Theorem (CST)

Knowing how different operations in an image or real space are connected to those in Fourier space is often beneficial. The central slice theorem establishes a link between an object's radon transformation and its two-dimensional Fourier transformation [66]. The theorem is as follows: the one-dimensional Fourier transformation of a projection at an angle of *θ* is the same as the radial or central slice at the same angle drawn from the object's two-dimensional Fourier domain. In order to illustrate this, we can write the two-dimensional Fourier transformation in terms of operators.

(8) $$\begin{array}{c} F_{2}O\left(r\right)=F_{1}RO\left(r\right). \end{array}$$

Another means in which the entity function can be reconstructed from its parallel representations is given by the central slice theorem. We take each projection's Fourier transformation and “position it” along the relevant radial slice. By running this step between 0 and *π* for all values of *θ*, the Fourier inversion helps one to recover the piece.

The article "Deep Learning-Based Image Reconstruction for Different Medical Imaging Modalities" was published in 2022. Journal: Comput Math Methods Med.

### 2.11. Filtered Back Projection (FBP)

One of the most prevalent techniques used in tomographic image restoration is the filtered back projection (FBP) algorithm. The method of estimating an object image slice of *f*(*x*, *y*) from a collection of projections *p*(*t*, *θ*) is image reconstruction. This role can be accomplished by many algorithms with various benefits. The basis of the image restoration mathematical kit is the [67] reconstruction algorithm. The FBP technique is commonly referred to as the convolution method for reconstructing a two-dimensional image using a one-dimensional integral equation. The most common reconstruction algorithm currently used in the application of CT is this method.

## 3. Databases

We give a comprehensive description of commonly utilized databases that are used for image reconstruction and segmentation. It should be noted that some of these works use information augmentation to increase the number of samples labelled, particularly those working with limited datasets. Increasing the amount of training samples by adding a transformation collection to the images helps to increase the data. Translation, reflection, rotating, warping, scaling, colour space flipping, cropping, and projections into key components are several common transformations. Data augmentation, particularly when learning from small databases, such as those in medical image analysis, has been shown to enhance the output of the models. It may also be helpful in having rapid integration, reducing the probability of overfitting, and increasing generalization. Data augmentation has shown to improve model efficiency by more than 20% for certain limited datasets. Most prominent medical image analysis databases with modalities and anatomic are shown in Figure 4.

### 3.1. Interstitial Lung Diseases (ILDs)

A digital series of interstitial lung disease (ILD) cases constructed at the University Hospitals of Geneva (HUG) would be made open to the public. The collection includes a high-resolution computed tomography (HRCT) image sequence of three-dimensional annotated areas of diseased lung tissue, as well as clinical criteria for individuals who have pathologically verified ILD diagnoses. Few samples of CT image slices in the ILD dataset for six lung tissue forms are shown in Figure 5. The library features 128 patients with one of 13 histological diagnoses of ILDs, 108 sequences of photographs of more than 41 litres of annotated lung tissue patterns, and a complete range of 99 ILD-related clinical criteria. On request and after signing of the licence agreement [68], the database is accessible for study.

The article "Deep Learning-Based Image Reconstruction for Different Medical Imaging Modalities" was published in 2022. Journal: Comput Math Methods Med.

### 3.2. Brain Tumour Segmentation (BraTS) Challenge

BraTS have typically focused on evaluating state-of-the-art techniques for the segmentation of brain tumours in multimodal magnetic resonance imaging (MMRI) data. In a workshop conducted as part of the MICCAI 2012 conference in October 2012 in Nice, France, the first benchmark was planned; then, this challenge dataset release was accessible in the 2013, 2015, 2017, 2018, and now 2020 BraTS challenge deadlines. Four MRI sequences are eligible for each patient in BraTS 2015: FLAIR, T1-C weighted, T1-weighted, and T2-weighted. The training sample includes 54 Low-Grade Gliomas (LGG) and 220 High-Grade Gliomas (HGG) from the BraTS 2015 challenge dataset [28]. BraTS 2017 focuses on segmenting inherently heterogeneous brain tumours, such as gliomas, using multi-institutional preoperative MRI imaging. BraTS 2017 also reflects on the estimation of patient overall survival rate [69] to assess the therapeutic significance of segmentation tasks. Multi-institutional preoperative MRI scans are used by BraTS 2019 and concentrate on segmenting intrinsically heterogeneous brain tumours, including gliomas. Sample MRI from the BraTS dataset are shown in Figure 6.

### 3.3. Alzheimer's Disease Neuroimaging Initiative (ADNI)

With the assistance of a public-private collaboration under the leadership of Dr. Michael W. Weiner, ANDI launched in 2004. ADNI's primary objectives are to evaluate more authentic and sensitive methods for multiple biomarkers such as MRI, Cat, structural magnetic resonance imaging (sMRI), and clinical examination to assess MCI development and early stages of AD. Second, the latest groundbreaking, unrestricted data-access programme was extended to all researchers worldwide. ADNI's original aim was to employ 800 people aged 55 to 90 years to enroll in the analysis of approximately 200 cognitively normal elderly individuals to be pursued for 3 years, 400 individuals to be followed for 3 years with MCI, and 200 individuals to be followed for two years with early AD. In the ADNI dataset MR images shown in Figure 7, the top row depicts the strength images, and the bottom row shows the manually segmented labeling.

The article "Deep Learning-Based Image Reconstruction for Different Medical Imaging Modalities" was published in 2022. Journal: Comput Math Methods Med.

### 3.4. MURA

MURA is a broad dataset of radio diagrams, including 14,863 upper extremity musculoskeletal tests. Each analysis involves one or more views and is manually labelled as either usual or abnormal by radiologists. A crucial rational radio challenge is to decide if a radiographic analysis is usual or abnormal: a study perceived as normal rules out illness and may remove the need for more medical tests or treatments for patients. The role of identifying musculoskeletal abnormality is especially important since more than 1.7 billion individuals worldwide are impaired by musculoskeletal conditions [70]. These disorders, with 30 million emergency room visits annually and growing, are the most prevalent source of serious, long-term pain and injury. An example from the MURA dataset is Towards Radiologist-Level Abnormality Identification in Musculoskeletal Radiographs shown in Figure 8. The MURA dataset comprises 9045 regular and 5818 irregular upper extremity musculoskeletal radiographic tests, covering the back, humerus, elbow, forearm, wrist, neck, and finger. One of the main public radiovisual picture datasets is MURA.

### 3.5. The Cancer Imaging Archive (TCIA)

TCIA is an extensive collection of cancer patient images available for public download. A large-scale lung cancer detection dataset for CT and PET/CT from the TCIA dataset is shown in Figure 9. The data are structured as “collections,” usually the imaging of patients linked to a particular condition, form or type of picture (CT, MRI, optical histopathology, etc.), or subject of study. The main file format used by TCIA for radiological imaging is DICOM. Ref. [71] also offers supporting image-related evidence such as medical results, care specifics, genomics, and expert analyses. Both users have links to most of the datasets in TCIA.

However, TCIA offers protection assistance to restrict, where necessary, access to datasets. For example, if a dataset needs to be exchanged for preliminary review amongst collaborators on TCIA, TCIA would facilitate this. The data provider may, at the time of request, provide the TCIA team with a list of partners that will have exclusive access. Getting the data mounted on TCIA will also enable the release of the data at a later date if needed.

### 3.6. Digital Database for Screening Mammography (DDSM)

The DDSM is a series of mammograms from the following organizations: the Massachusetts General Hospital, the School of Medicine at Wake Forest University, the Holy Heart Hospital, and the St. Louis School of Medicine at Washington University. The DDSM was created with funding from the Department of Defense Breast Cancer Research Program and the US Army Research and Material Command, and the DDSM's principal designers obtained the appropriate patient permissions. The instances include calcification and bulk ROIs, as well as the following details that may be beneficial for CADe and CADx algorithms: descriptors for mass form, mass margin, type of calcification, distribution of calcification, and breast density from the Breast Imaging Reporting and Data System (BI-RADS); BI-RADS overall rating from 0 to 5; and abnormality subtlety ranking from 1 to 5. An example of annotated mammogram images from DDSM database is shown in Figure 10.

The article "Deep Learning-Based Image Reconstruction for Different Medical Imaging Modalities" was published in 2022. Journal: Comput Math Methods Med.

### 3.7. Open Access Series of Imaging Studies (OASIS)

In the Open Access Sequence of Imaging Research (OASIS), OASIS-3 is the current publication aimed at rendering neuroimaging databases widely accessible to the science community. They hope to encourage potential developments in fundamental and clinical neuroscience by compiling and freely distributing this multimodal dataset produced by the Knight ADRC and its associated studies. For hypothesis-driven data analyses, neuroanatomical atlas creation, and segmentation algorithm development, previously published data for OASIS-Cross-sectional and OASIS-Longitudinal was used. For natural ageing and Alzheimer's disease [72], OASIS-3 is a longitudinal neuroimaging, behavioral, emotional, and biomarker dataset. Sample images from the OASIS dataset are shown in Figure 11. OASIS databases (Central.xnat.orgs) provide the population with free access to a vast collection of neuroimaging and processed imaging evidence across a diverse demographic, cognitive, and genetic continuum, as well as a readily available forum for neuroimaging, clinical, and cognitive studies on natural ageing and cognitive impairment. Any of the data can be obtained from http://www.oasis-brains.org/.

### 3.8. Autism Brain Imaging Data Exchange (ABIDE)

Autism spectrum disorder (ASD) is defined by qualitative dysfunction and by repeated, restrictive, and stereotyped behaviors/interests in social reciprocity. ASD is now known to occur in more than 1% of infants, which was historically considered uncommon. Their speed and therapeutic effects have not kept up with the urgency to find forms of assessing disease at younger ages, choosing appropriate therapies, and forecasting performance, amid ongoing scientific advancements. This is mainly because of the ambiguity and variability of ASD. Large-scale samples are required to face these obstacles, but single labs are unable to collect enough large datasets to expose the brain structures underlying ASD. In response, to accelerate our knowledge of the neurological basis of autism, the Autism Brain Imaging Research Sharing (ABIDE) project has aggregated functional and structural brain imaging data obtained from laboratories across the globe. The ABIDE project currently comprises two large-scale collections: ABIDE I and ABIDE II, with the overall aim of promoting discovery science and sample-to-sample comparisons.

The article "Deep Learning-Based Image Reconstruction for Different Medical Imaging Modalities" was published in 2022. Journal: Comput Math Methods Med.

The selection was created by combining datasets gathered from more than 24 different foreign brain imaging institutions and made available to researchers all around the world. An example of the ABIDE dataset which applied a pipeline to an input volume to prepare it for feature extraction is shown in Figure 12.

### 3.9. OpenNeuro

OpenNeuro is a directory of open neuroimaging data [73]. The data is shared under a Creative Commons CC0 licence, which provides researchers as well as community scientists with a large variety of brain imaging data. The database relies mainly on results from practical magnetic resonance imaging (fMRI) but also encompasses other modalities of imaging, including longitudinal and diffusion MRI, electroencephalography (EEG), and magnetoencephalography (MEG). Open fMRI is a collaboration of Stanford University's Centre for Reproducible Neuroscience. An example of brainstem MRI from the OpenNeuro dataset is shown in Figure 13. The National Science Foundation, the National Institution on Mental Health, the National Institute on Substance Addiction, and the Laura and John Arnold Foundation also supported the creation of the OpenNeuro resource.

### 3.10. Osteoarthritis Initiative (OAI)

The Osteoarthritis Initiative (OAI), supported by the National Institutes of Health, is a multicenter, ten-year retrospective analysis of men and women. The OAI's aims are to include tools to allow a deeper understanding of knee osteoarthritis prevention and care, one of the most prevalent causes of adult impairment. The supervised machine learning phase of AQ-CART employed a training dataset of 378 patient single-knee MRI images as input data. These were chosen to reflect the full spectrum of structural severity of radiographic OA, like Kellgren-Lawrence medial compartment grades 0-4, OA lateral compartment, along with good young knees that appear to have thicker cartilage. An OAI 3D double-echo-in-steady-state sequence was used to capture the 286 images (DESS-we) [74]. A sample of knee MRI from the Osteoarthritis Initiative (OAI) dataset is shown in Figure 14.

### 3.11. Ischemic Stroke Lesion Segmentation (ISLES)

Over the past three years (2015, 2016, and 2017), this challenge for stroke lesion segmentation has been very common and has culminated in several approaches that help to overcome major challenges in contemporary stroke imaging research. Many activities include medical image processing, for which innovative approaches are constantly proposed. Varying dataset size and heterogeneity, though, render it virtually difficult to fairly equate numerous approaches. Challenges such as ISLES seek to address these limitations and establish a shared structure for adequate comparison of outcomes by delivering a high-quality data collection publicly and predefined assessment guidelines. A sample of ischemic lesion segmentation in multispectral MR images is shown in Figure 15.

The article "Deep Learning-Based Image Reconstruction for Different Medical Imaging Modalities" was published in 2022. Journal: Comput Math Methods Med.

The data collection for training comprises 63 patients. In certain hospital instances, the stroke lesion has two slabs to protect. There are brain areas that are pre-, or partially, overlapping. For the first and second slabs, slabs per patient are indicated with the letters “A” and “B.” In SMIR, mapping is also given between case number and training term. A test range consisting 40 stroke cases [74] would assess proven techniques.

### 3.12. Automated Cardiac Diagnosis Challenge (ACDC)

From real clinical examinations acquired at the University Hospital of Dijon, the total ACDC dataset was developed. Acquired knowledge was thoroughly anonymized and handled in compliance with the rules laid down by the Dijon Hospital Local Ethics Committee (France). Our dataset encompasses many well-defined pathologies with ample cases to (1) train machine learning methods adequately and (2) test explicitly the variations of the key physiological parameters obtained from cine-MRI (in particular, diastolic volume and ejection fraction).

As mentioned below, the dataset consists of 150 assessments (all from separate patients) grouped into 5 equally distributed subgroups (4 pathological groups + 1 balanced topic group). In addition, the following additional details come for each patient: weight, height, as well as the instants of the diastolic and systolic processes. After personal enrollment, the database is made accessible to the participants by means of two datasets from the designated online assessment website: (i) a study dataset of 100 patients along with the relevant manual references focused on the review of one professional expert; (ii) a test dataset consisting of 50 new patients, without manual notes, but with the above patient details. Via the NIfTI format, raw input images are given. An example of MRI from the ACDC challenge dataset is shown in Figure 16.

## 4. Performance Evaluation

We include a description of some of the common metrics used in assessing the segmentation algorithm output in this portion. In different ways, such as quantitative precision, speed, and storage specifications, the algorithm should be tested. Much of the research work to date focuses on the metrics used to determine the accuracy of the model.

The article "Deep Learning-Based Image Reconstruction for Different Medical Imaging Modalities" was published in 2022. Journal: Comput Math Methods Med.

### 4.1. Precision/F1 Score/Recall

They are standard metrics for reporting the accuracy of several models of classical image segmentation. For each class, as well as at the aggregate level, precision and recall may be described as follows:

(9) $$\begin{array}{c} \text{Precision}=\frac{\text{TP}}{\text{TP}+\text{FP}},\\ \text{Recall}=\frac{\text{TP}}{\text{TP}+\text{FP}}, \end{array}$$

where TP refers to the true positive fraction, the false positive fraction is referred to by FP, and the false negative fraction is referred to by FN. We are generally interested in a blended version of precision and rates of recall. A common metric of this kind is called the F1 score, which is defined as the harmonic mean of consistency and recall:

(10) $$\begin{array}{c} \text{F}1\text{ score}=\frac{2\text{PrecRec}}{\text{Prec}+\text{Rec}}. \end{array}$$

### 4.2. Dice Coefficient

Another popular metric for image segmentation is the Dice coefficient, and it is more widely used in medical image analysis.

(11) $$\begin{array}{c} \text{Dice}=\frac{2\text{TP}}{2\text{TP}+\text{FP}+\text{FN}}=\text{F}1. \end{array}$$

### 4.3. Jaccard Index or Intersection over Union (IoU)

It is one of the most widely used semantic segmentation metrics. The area of intersection between the forecast segmentation map and the ground truth is defined as divided by the area of union between the forecast segmentation map and the ground truth:

(12) $$\begin{array}{c} \text{IoU}=J\left(A,B\right)=\frac{J\cap B}{J\cup B}, \end{array}$$

where, respectively, *A* and *B* denote the ground truth and the projected segmentation maps. It has a scale of 0 to 1. This section is concluded with the important discussion about the above-mentioned metrics. We have seen that in most experiments, IoU is used for detection and the Dice coefficient is used for segmentation tasks. As a loss function, the Dice coefficient is used because it is distinguishable in segmentation tasks where IoU is not distinguishable. Both can be used to measure the efficiency of your model as a metric, but only the Dice coefficient is used as a loss function. Owing to the overwhelming number of class events, the class imbalance dilemma is a common problem concerning machine learning.

## 5. Challenges and Future Directions

While deep learning-based models continue to dominate medical imaging, there are still plenty of deep modelling challenges that restrict the application and adoption in the clinical practice of these new approaches. These problems are often posed to researchers working in similar fields as future ideas. In order to create new deep models in diagnostic imaging, there is only minimal labelled data available. Medical image transcription is time intensive and allows physicians to have deep knowledge. Can we build efficient models of learning that could really facilitate efficient use of both labelled and unlabeled data?

The article "Deep Learning-Based Image Reconstruction for Different Medical Imaging Modalities" was published in 2022. Journal: Comput Math Methods Med.

It is typically difficult to collect very huge health-care data for a particular task due to morbidity and privacy issues. In addition, (by definition) the number of rare cases is limited but can be more significant than common cases. To effectively extract information from these small samples and recognize such unequal value among the samples, can we design learning models and data augmentation techniques? The clinical judgement is not focused exclusively on images by radiologists. In decision-making, more input from the patients and the experience of the doctors from their years of medical school training are also important. In order to improve system performance, it is therefore necessary to incorporate data gathered from various different sources into deep modelling. Reasoning is almost as crucial as, if not even more essential than, referring. Most deep models currently mask the cognitive development. There is a possibility that the model makes predictions based on inaccurate logic. It renders the model unstable. Can deep simulation be integrated with logic or a graph of medical expertise? This will further decrease the amount of labeled images that will be needed to train deep learning models without losing output.

## 6. Conclusion

A study of the latest literature on deep learning for medical imaging has been presented in this article. A detailed review of the image reconstruction methods and concise description of the components has been presented. A summary of some of the most widely used datasets for MR image reconstruction is given in the third part of this article. The key problems facing deep learning in medical image processing were identified in the later section of the paper; also, the possible directions for overcoming these challenges were discussed. Presented literature will exploit huge advantages for medical imaging applications and will boost the ability of artificial algorithms to assist radiologists.

## Figures and Tables

**Figure 1:** MRI system view.

**Figure 2:** Summary of data from the European Union (EU) on the use of imaging equipment and number of magnetic resonance imaging scans (2019).The indicator is provided in the form of total value and position. The measurement is per 1000 inhabitants.

The article "Deep Learning-Based Image Reconstruction for Different Medical Imaging Modalities" was published in 2022. Journal: Comput Math Methods Med.

**Figure 3:** Conventional image reconstruction method flow chart.

**Figure 4:** Most prominent medical image analysis databases with modalities and anatomic.

**Figure 5:** Few samples of CT image slices in the ILD dataset for six lung tissue forms [46].

**Figure 6:** Example MRI from BraTS dataset.

**Figure 7:** The ADNI dataset MR images: (a) depicts the strength images, and (b) shows the manually segmented labeling.

**Figure 8:** An example from the MURA dataset is Towards Radiologist-Level Abnormality Identification in Musculoskeletal Radiographs.

**Figure 9:** A large-scale lung cancer detection dataset for CT and PET/CT from the TCIA dataset.

**Figure 10:** Annotated mammogram images from DDSM database.

**Figure 11:** Sample images from OASIS dataset.

**Figure 12:** An example of ABIDE dataset on which a pipeline was applied to an input volume to prepare it for feature extraction.

**Figure 13:** Brainstem MRI from OpenNeuro dataset.

**Figure 14:** A sample of knee MRI from Osteoarthritis Initiative (OAI) dataset.

**Figure 15:** A sample of ischemic lesion segmentation in multispectral MR images.

**Figure 16:** Example of MRI from ACDC challenge dataset.

**Table 1:** Medical image reconstruction techniques.

Methodologies applied	Performance	Drawbacks
Analytical methods	They are efficient.	Requires proper sampling.
Iterative methods	The imaging device's statistical and physical features are considered.	Inhomogeneous magnetic fields, for example, cause differences between the model and physical variables.
Learning-based and data-driven methods	Learned signal models can be used to rebuild images from low-quality data.	They are inefficient in terms of computing and necessitate enormous amounts of training data.

**Table 2:** A summary of articles that use deep learning approaches for image reconstruction in MRI.

Reference	Brief overview
[37]	A DNN model for image reconstruction from subsampled MRI scans. It can also be used for image denoising and super-resolution. However, not all image properties are explicitly exploited.
[38]	A deep learning framework for MR image reconstruction called AUTOMAP. It is accurate when compared to conventional methods. However, it is computationally intensive.
[39]	From significantly undersampled *k*-space data, a CNN framework for high-quality cardiovascular MR image reconstruction.
[40]	A model that blends variational model mathematics with deep learning. Standard reconstruction techniques are outperformed by the model. There is further work to be done on several types of error measures.
[23]	A DNN-based technique for MR image reconstruction. In the weighted loss function, smaller weights are assigned to noisy training images.
[41]	For rapid and accurate CS-MRI reconstruction, a deep learning model has been developed. There is still a requirement to comprehend the proposed method's design.
[42]	A framework for reconstructing MR images from *k*-space data that has been undersampled. The structure is also noise-resistant.
[25]	A method for image reconstruction denoising and data integrity enforcement. Due to a decrease in trainable parameters, it does not need a large amount of training data.
[43]	A deep neural network-based image reconstruction model. The computational difficulty of compressed sensing-based approaches was addressed in the model.
[44]	A complete framework for high-resolution MR reconstruction. From noisy, low-resolution clinical MRI data, good-quality pictures are recreated.

The article "Deep Learning-Based Image Reconstruction for Different Medical Imaging Modalities" was published in 2022. Journal: Comput Math Methods Med.

**Table 3:** A summary of articles that use deep learning approaches for image reconstruction in CT.

Reference	Brief overview
[46]	A model based on Wasserstein generative adversarial networks for 2D CT slice image reconstruction from a small number of prediction images. Expert radiologists must confirm the model's accuracy.
[47]	A U-net-based image reconstruction framework. It is superior to noise and angle artefacts in terms of visual structure preservation, but it is computationally costly and requires large training datasets.
[48]	A more relaxed variant of projected gradient descent (PGD) is used in this model. The results demonstrate that the new technique outperforms the previous one.
[49]	An approach for CT image reconstruction based on deep learning. When compared to other state-of-the-art approaches, the results show enhanced image quality with less image noise.
[50]	A lightweight framework for a few-view CT reconstruction approach. It learns an end-to-end mapping between a few-view picture optimization and a full-view image optimization.
[51]	For high-quality CT reconstructions, a deep learning architecture was developed. The framework is capable of distinguishing and removing noise from the input signal.
[52]	Iterative reconstructions of data from genuine CT systems using a TensorFlow framework. The drawback is that it necessitates the use of graphics processing units (GPUs).
[53]	During reconstruction, a CNN framework is used to remove streaks from CT images. To discriminate between objects and characteristics, the framework requires further training.
[54]	A deep learning model for reconstructing high-quality images from sinogram data. It reduces noise, improves spatial resolution, and is quick without sacrificing quality.
[55]	For CT reconstruction, there is a framework called LEARN. It boosts image quality as well as computational efficiency. The framework still has to be optimized for clinical applications.

The article "Deep Learning-Based Image Reconstruction for Different Medical Imaging Modalities" was published in 2022. Journal: Comput Math Methods Med.

**Table 4:** A summary of articles that use deep learning approaches for image reconstruction in other modalities.

Reference	Brief overview
[56]	Wave flow is a deep learning-based tool. The technology was evaluated using data acquired from wire and cyst phantoms. Both GPU and CPU are supported by the tool.
[57]	For ultrasound image reconstruction, a generative adversarial network (GAN) framework was developed. The suggested framework produced higher-quality ultrasound reconstructions.
[58]	A method for faster B-mode ultrasound imaging. When compared to other current approaches, PSNR, CNR, and SSIM all increased significantly.
[59]	PET image reconstruction using an encoder-decoder system. The use of synthetic data rather than genuine patient data is a drawback.
[60]	To overcome the mismatch of noise levels, a framework for iterative PET reconstruction employing denoising CNN and a local linear fitting function has been developed. It beats traditional approaches in terms of total variation.
[30]	In electromagnetic tomography, a strategy for resolving imaging difficulties has been developed (EMT). Its practicality has been confirmed by preliminary results.
[61]	A diffuse optical tomography (DOT) projection data-based image reconstruction model. Validation of the model clinical situations is required.
[40]	In optical microscopy, the work offered an overview of DNNs. DNNs increase the quality of image reconstruction in optical microscopy, according to the findings.

**Table 5:** Major IR algorithm classifications based on function mechanism, including product names, vendors, and acronyms.

Algorithms	Acronym	Vendor	Recons type
ASIR	Adaptive statistical iterative reconstruction	GE Healthcare, Milwaukee, MI	Hybrid
SAFIRE	Sinogram-affirmed iterative reconstruction	Siemens Healthcare, Forchheim, Germany	Hybrid
AIDR 3D	Adaptive iterative dose reduction 3D	Toshiba Medical Systems, Japan	Hybrid
IMR	Iterative model reconstruction	Philips Medical Systems	Pure
iDOSE4	Product name	Philips Medical Systems, Best, Netherlands	Pure
IRIS	Iterative reconstruction in image space	Siemens Healthcare, Germany	Hybrid
AMIR	*Advanced modeled iterative reconstruction*	Siemens, Germany	Hybrid
MBIR	Model-based iterative reconstruction	GE Healthcare	Hybrid
Safe CT	Product name	Medic Vision	Image based
